The article "Identification of the Ferroptosis-Associated Gene Signature to Predict the Prognostic Status of Endometrial Carcinoma Patients" was published in 2021. Journal: Comput Math Methods Med.

# Identification of the Ferroptosis-Associated Gene Signature to Predict the Prognostic Status of Endometrial Carcinoma Patients

**DOI:** 10.1155/2021/9954370

**Published:** 2021-09-07

**Authors:** Jinlong Qin, Xiaowen Shao, Lei Wu, Hongling Du

**Affiliations:** ^1^Department of Obstetrics and Gynecology, Putuo People's Hospital, Tongji University School of Medicine, Shanghai, China; ^2^Department of Obstetrics and Gynecology, Shanghai Tenth People's Hospital, Tongji University School of Medicine, Shanghai, China; ^3^Department of Anesthesiology, Putuo People's Hospital, Tongji University School of Medicine, Shanghai, China

## Abstract

Endometrial carcinoma (EC) is one of the most common gynecological carcinomas. As previously described, ferroptosis was reported to exhibit a significant association with the development of malignant neoplasms. Nevertheless, there are few studies towards the association between the implication of ferroptosis-related genes (FRGs) and the prognostic status of patients with EC. Our study demonstrated that ferroptosis-related genes were evidently differently expressed in EC. Further analysis showed that SLC7A11, SAT1, CDKN1A, and TP5MC3 expression was linked to the low stage, grade of pTNM, and longer survival time. Bioinformatics analysis demonstrated that these ferroptosis-related regulators played a crucial role in EC by modulating multiple biological processes, such as cell cycle, citrate cycle (TCA cycle), metabolism-related pathways, ERK activation, p53 signaling pathway, cellular senescence, TAp63 pathway, and Notch signaling pathway. Of note, our results showed that ATP5MC3, CDKN1A, and SLC7A11 expression was dramatically positively related with the tumor mutational burden (TMB) score in EC. However, we did not observe a significant correlation between SAT1 and the TMB score in EC. These findings for the first time demonstrated that ferroptosis was displayed crucially in EC progression. We speculated that our findings offered novel targets and strategies for personalized treatment.

## 1. Introduction

Uterine corpus endometrial carcinoma (UCEC) is one of the commonly occurring endometrial carcinomas (EC) [1], which is a malignant endometrial epithelial carcinoma in women and accounts for about 80% amid adenocarcinomas [2]. Endometrioid adenocarcinoma occupied 80% amongst overall EC and was thought to be estrogen-dependent type I EC [3]. Serous endometrial carcinomas are generally referred to be type II of estrogen-independent cancer [4]. As global carcinoma statistics has shown, about 382000 new EC cases were produced worldwide, accompanied with almost 90000 death tolls in 2018 [5]. In the past five years, there were several studies showing that EC took up 20%–30% of female genital tract malignancies and the occurrence ratio of EC is growing [6, 7]. In the United States, the lethality ratio of EC is the highest in female and the occurrence proportion of EC is elevating [8]. In 2017, 61380 women in the United States were diagnosed with EC and 10920 women died of EC [9]. The five-year cause-specific survival rate for serous cancer is 43%, while those for endometrioid, mucinous, and clear cell carcinoma are 82%, 71%, and 66% respectively [9]. 20% to 30% of patients with EC are diagnosed with the advanced stage in the process of surgery. It is estimated that the five-year survival rate of patients in stage III ranged from 40% to 70% and was within 0 to 10% in stage IV. Herein, to determine efficacious biomarkers and therapeutic targets for predicting and ameliorating the prognostic status of EC patients is essential.

The article "Identification of the Ferroptosis-Associated Gene Signature to Predict the Prognostic Status of Endometrial Carcinoma Patients" was published in 2021. Journal: Comput Math Methods Med.

Ferroptosis, displaying a close relationship with the metabolism of amino acids, iron, and polyunsaturated fatty acids and the biosynthesis of glutathione, phospholipids, and NADPH is a new discovery form of cell death with the characteristics of iron-dependent lipid peroxidation [10, 11]. Ferroptosis is another type of programmed necrotic cell death that participates in the process of iron-dependent lipid peroxidation [12, 13]. Iron chelator, lipid peroxidation inhibitor, and reduced intracellular polyunsaturated fatty acids can inhibit ferroptosis [14]. There is increasing evidence showing that a link existed in ferroptosis and the pathophysiological development of neurological diseases, comprising stroke, degenerative diseases, neurotrauma, and carcinoma [15]. Ferroptosis is related to the treatment of carcinomas [16]. Initial data suggested that ferroptosis can inhibit the growth and development of neoplasms and may be beneficial for the treatment of carcinomas [17]. Among neoplasms, ferroptosis facilitates the mobility and invasion of tumor cells and induces the progression and metastasis of carcinomas, making them resistive to drugs against neoplasms [18]. Presently, some reports have revealed that lots of molecular modulators were associated with ferroptosis and human carcinoma development, including EC [19]. For instance, miR-522 secreted by cancer-associated fibroblasts (CAFs) resulted in a suppression of ferroptosis but induced acquired chemical resistance in gastric cancer [19, 20]. Cytochrome P450 oxidoreductase (POR), demonstrating inherent and induced susceptibility to ferroptosis, was shown to be essential for ferroptotic cell death in carcinomas [20]. CD8^+^ T cells modulated ferroptosis of neoplasms in cancer immunotherapy [21]. ALOX12 is necessary for p53-mediated tumor inhibition by a unique pathway of ferroptosis [22]. However, the expression profile and molecular ferroptosis regulators in EC remained largely unclear.

The article "Identification of the Ferroptosis-Associated Gene Signature to Predict the Prognostic Status of Endometrial Carcinoma Patients" was published in 2021. Journal: Comput Math Methods Med.

Nevertheless, little is known about the relationship between the signification of ferroptosis-associated genes (FRGs) and the prognostic status of patients with EC. Herein, our study here systematically explored the relationship utilizing The Cancer Genome Atlas (TCGA) database. Our findings were conducive to better evaluate patients' prognosis and offered a new perspective for the treatment of individualized EC patients.

## 2. Materials and Methods

### 2.1. Clinical Information and mRNA Expression Dataset of Patients

Ferroptosis-related genes were obtained from The Human Genome Database (https://www.genecards.org/) by searching the keywords “Ferroptosis” and other related literatures [11, 23]. The mRNA expression profiles of 543 EC samples and 23 normal samples from TCGA were extracted. The clinical information of EC patients was comprised of age, grade, AJCC stage, histologic type, overall survival (OS), and disease-free survival (DFS).

### 2.2. To Identify and Analyze the Differentially Expressed FRGs (DEFRGs)

The limma package [24] was employed to determine the DEFRGs in 1184 FRGs between EC tissues and normal tissues and visualize their expression by volcano plots and heatmaps. The significant threshold indicated a false discovery rate < 0.05 and ∣logFC | >1. Then, based on the selected DEFRGs, we conducted Gene Ontology (GO) and Kyoto Encyclopedia of Genes and Genomes (KEGG) pathway enrichment analyses. What is more, the STRING database was employed to establish a protein–protein interaction (PPI) network among the selected genes and further validate the association between the DEFRGs. The minimum required interaction indicated score was 0.4. The hub genes indicated the genes with a node degree > 15.

### 2.3. To Construct and Analyze the Implication of Prognosis

Univariate Cox regression analysis was conducted to define the prognostic value of the DEFRGs and verify the OS, PFS, and DFS in EC patients with these DEFRGs. In order to prevent collinearity, LASSO analysis was employed [25]. To explore the prognostic implication of FRG, multivariable Cox analysis was taken.

On the basis of the average risk score, we separated EC patients into two groups: high- and low-risk groups. For comparison of the prognostic differences existing in two different groups, we conducted Kaplan–Meier (K-M) survival curves and the log-rank test. Besides, we counted receiver operating characteristic (ROC) curves to assess the difference of the prognostic model.

### 2.4. Bioinformatics Analysis

The raw number of RNA-sequencing data (level 3) and corresponding clinical information from XX were acquired from TCGA dataset (https://portal.gdc.cancer.gov/) in January 2020. The acquisition and application of all methods were in line with the protocol and principles.

The article "Identification of the Ferroptosis-Associated Gene Signature to Predict the Prognostic Status of Endometrial Carcinoma Patients" was published in 2021. Journal: Comput Math Methods Med.

Sanguini diagram was built based on the R software package ggalluvial. All the above analysis methods and R package were implemented by R foundation for statistical computing (2019), version 4.0.3, *P* < 0.05.

The R software package ConsensusClusterPlus (v1.54.0) was applied for consistency analysis [26]. The maximum number of clusters is 6, and 80% of the total sample is drawn 100 times, clusterAlg = ^“^hc,^”^ innerLinkage = ^“^ward.D2.” Use the R software package pheatmap (v1.0.12) for clustering heat maps. The gene expression heatmap retains genes with SD > 0.1. If the number of input genes is more than 1000, it will extract the top 25% genes after sorting the SD.

## 3. Results

### 3.1. Gene Expression of Ferroptosis Modulators in the Development of EC

We evaluated the transcriptome profile of ferroptosis modulators in details. We downloaded RNA-Seq data from TCGA-UCEC cohorts, containing the data of carcinoma tissue (*n* = 499) and paracarcinoma tissue (*n* = 52). The detail of ferroptosis modulators was picked up and used for the DEG analysis.  Figure 1 shows that all the ferroptosis modulators were differently expressed in UCEC samples compared to those in normal tissues. Among them, HSPA5, HSPB1, CS, CARS, EMC2, TFRC, NCOA4, ACSL4, RPL8, GPX4, CDKN1A, LPCAT3, NFE2L2, CISD1, SLC1A5, SAT1, FDFT1, and MT1G were significantly overexpressed in grades 1 to 3 of tumor samples compared to normal tissues. However, FANCD2, SLC7A11, GLS2, DPP4, and ALOX15 were obviously suppressed in grades 1–3 of tumor samples compared to normal tissues.

### 3.2. Identification of Interaction among Ferroptosis-Related Regulators in EC Development

In order to explore the interaction among ferroptosis-related regulators in EC, we calculated the correlation among them.  Figure 2(a) revealed that most of ferroptosis modulators displayed an association with each other. Our data suggested that HSPB1, CS, CARS, EMC2, NCOA4, ACSL4, GPX4, CDKN1A, LPCAT3, NFE2L2, CISD1, SLC1A5, FDFT1, MT1G, FANCD2, SLC7A11, GLS2, DPP4, and ALOX15 expression exhibited a positive correlation with other modulators. The opposite correlation was demonstrated between HSPA5 and ATP5MC3 and other modulators. Meanwhile, some regulators such as TFRC, SAT1, and RPL8 exhibited a poor association with others.

The PPI network of ferroptosis modulators showed that GLS2, SLC1A5, SLC7A11, GPX4, ALOX15, NFE2L2, CDKN1A, SAT1, ACSL4, and LPCAT3 had the potential to interplay with each other (Figure 2(b)). Meanwhile, EMC2, ATP5MC3, RPL8, CARS, TFRC, and DPP4 formed a PPI network and HSPB1, CS, and HSPA5 formed a PPI network (Figure 2(b)). Notably, no connection was shown between CISD1, FANCD2, FDFT1, LPCAT3, MT1G, and NCOA4 and other modulators (Figure 2(b)).

The article "Identification of the Ferroptosis-Associated Gene Signature to Predict the Prognostic Status of Endometrial Carcinoma Patients" was published in 2021. Journal: Comput Math Methods Med.

### 3.3. Identification of DEFRGs Associated with Prognosis in EC Development

Then, we assessed whether ferroptosis-related regulator expression exhibited a relationship with EC prognosis.  Figure 3 suggested that a higher expression level of CDKN1A (Figure 3(a)), SLC7A11 (Figure 3(b)), and SAT1 (Figure 3(c)) displayed a positive relationship with longer DFS time. Nevertheless, highly expressed ATP5MC3 led to shorter DFS time in EC (Figure 3(d)).

We calculated each patient's risk score. Through the “survminer” R package, we obtained the median cutoff points of ATP5MC3, SAT1, SLC7A11, and CDKN1A and classified patients into the high-risk group (*n* = 176) and low-risk group (*n* = 177) (Figures 4(a)–4(d)). The KM survival curves further confirmed that highly expressed ATP5MC3 gave rise to shorter DFS time in EC (Figure 4(e)). In addition, higher expression levels of CDKN1A, SLC7A11, and SAT1 were positively related to longer DFS time (Figures 4(f)–4(h)). To evaluate the predictive efficiency of CDKN1A, SLC7A11, SAT1, and ATP5MC3 in the 1-, 3-, and 5-year survival ratio, we carried out a ROC curve analysis. The area under the ROC curve (AUC) of ATP5MC3 was 0.655 at 1 year, 0.672 at 3 years, and 0.668 at 5 years (Figures 4(i)–4(l)). The area under the ROC curve (AUC) of SAT1 was 0.684 at 1 year, 0.674 at 3 years, and 0.627 at 5 years, individually. The area under the ROC curve (AUC) of SLC7A11 was 0.539 at 1 year, 0.574 at 3 years, 0.579 at 5 years, and that of CDKN1A was 0.69 at 1 year, 0.625 at 3 years, and 0.59 at 5 years (Figures 4(i)–4(l)).

We next calculated the correlation between FRGs' expression and overall survival time by dividing EC patients into ATP5MC3, SAT1, SLC7A11, and CDKN1A high and low groups (Figures 5(a)–5(d)). The higher expression levels of CDKN1A, SLC7A11, and SAT1 and lower expression of ATP5MC3 were positively related to longer DFS time (Figures 5(f)–5(h)). The KM survival curves further confirmed this finding. To evaluate the predictive efficiency of CDKN1A, SLC7A11, SAT1, and ATP5MC3 in the 1-, 3-, and 5-year OS ratio, we carried out a ROC curve analysis. The areas under the ROC curve (AUC) of ATP5MC3, SAT1, SLC7A11, and CDKN1A were also determined (Figures 5(i)–5(l)).

### 3.4. The expression of ferroptosis-related regulators was differently expressed in the development of EC.

We further confirmed the expression levels of SLC7A11, SAT1, CDKN1A, and TP5MC3 in EC and normal samples by combining the TCGA database and GTEX database with GEPIA. Our results demonstrated that SLC7A11, SAT1, and TP5MC3 were also upregulated in EC compared to normal samples. However, CDKN1A was deceased in EC compared to normal samples (Figures 6(a)–6(d)). Then, we determined ferroptosis-related regulator expression and clinical characteristics in EC development, including the pTNM_stage, grade, and survival status. We found that high expression of SLC7A11 (Figure 6(e)), CDKN1A (Figure 6(f)), and SAT1 (Figure 6(h)) was linked to low pTNM_stage, grade, and longer survival time. However, overexpression of TP53MC3 was associated with advanced pTNM_stage, grade, and shorter survival time in EC (Figure 6(g)). All the results were in line with the above analysis and indicated that SLC7A11, SAT1, and CDKN1A may serve as tumor suppressors and TP53MC3 was a probable oncogene in EC.

The article "Identification of the Ferroptosis-Associated Gene Signature to Predict the Prognostic Status of Endometrial Carcinoma Patients" was published in 2021. Journal: Comput Math Methods Med.

### 3.5. The Expression of Ferroptosis-Related Regulators Presented an Association with the TMB Score in EC Development

Previous studies demonstrated that mutational load of neoplasm provided a prediction of survival after immunotherapy across multiple types of carcinoma [27–29]. Here, our study attempted to determine the correlation between ferroptosis-related regulators and TMB score in EC. The results showed that ATP5MC3 (Figure 7(a)), CDKN1A (Figure 7(b)), and SLC7A11 (Figure 7(c)) were significantly positively associated with the TMB score in EC. However, we did not observe a significant correlation between SAT1 and the TMB score in EC (Figure 7(d)). These results suggest that ATP5MC3, CDKN1A, and SLC7A11 may serve as a predictive marker of immunotherapy in EC.

### 3.6. Bioinformatics Analysis of Ferroptosis-Associated Regulators in EC

For in-depth analysis of the functions and pathways of SLC7A11, SAT1, CDKN1A, and ATP5MC3, we conducted GO analysis and KEGG pathway enrichment analysis accordingly. Our results showed that ATP5MC3 was related to regulate spliceosome, proteasome, cell cycle, and citrate cycle (TCA cycle) (Figure 8(a)). SLC7A11 was found to be related to multiple metabolism-related pathways (such as sodium-coupled phosphate cotransporters, chondroitin sulfate/dermatan sulfate metabolism, chondroitin sulfate biosynthesis, glyoxylate metabolism, serotonin, and melatonin biosynthesis) and ERK activation (Figure 8(b)). CDKN1A was involved in regulating the p53 signaling pathway, cellular senescence, and VEGF signaling pathway (Figure 8(c)). In addition, our results showed SAT1 was related to the activation of multiple signaling, such as AKT phosphorylation of cytosolic targets, TP53 network, TAp63 pathway, hypoxia, and p53 in the cardiovascular system, cell cycle: G2/M checkpoint, and Notch signaling pathway (Figure 8(d)).

The article "Identification of the Ferroptosis-Associated Gene Signature to Predict the Prognostic Status of Endometrial Carcinoma Patients" was published in 2021. Journal: Comput Math Methods Med.

## 4. Discussion

Recently, there is growing evidence showing that ferroptosis exhibited a close relationship with the development, metastasis, and drug resistance of carcinoma [30, 31]. Several studies had revealed that the differently expressed genes were correlated with the prognosis of human cancers. For example, ACSL4 is a predictive biomarker of sorafenib sensitivity in hepatocellular carcinoma [32]. ACSL4 suppresses glioma cell proliferation via activating ferroptosis [33]. GLS2 is protumorigenic in breast cancers [34]. GPX4 and GPX7 were overexpressed in the tissues of human hepatocellular carcinoma [35]. Hypermethylation of MT1G is associated with the higher stage of tumor in EC [36]. NFE2L2 is reported to be a prospective biomarker for prognosis and is shown to be related with immune infiltration in brain lower-grade glioma [37]. Mutations of NFE2L2/KEAP1 was correlated with higher TMB value/PD-L1 expression and powerfully ameliorated clinical outcome with the use of immunotherapy [38]. Moreover, the signature of FRG could indicate cell death of glioma and the progression of glioma patients [39] and the OS in hepatocellular cancer patients [40]. However, the expression profile and molecular ferroptosis regulators in EC remained largely unclear. The present study for the first time showed that all of ferroptosis regulators were differently expressed in UCEC samples compared to normal tissues. Further analysis showed that ferroptosis-related regulators were positively correlated with other regulators. Bioinformatics analysis demonstrated that these ferroptosis-related regulators played a crucial role in EC by modulating multiple biological processes, such as cell cycle, citrate cycle (TCA cycle), metabolism-related pathways, ERK activation, p53 signaling pathway, cellular senescence, TP53 network, TAp63 pathway, and Notch signaling pathway.

Over the past decades, emerging studies demonstrated that the regulation of multiple biological processes such as biological signal transmission, gene expression regulation, energy and material metabolism, and cell cycle regulation depends on protein-protein networks, not a single protein [41, 42]. In this study, we calculated the correlation among FRGs to explore the interaction among ferroptosis-related regulators in EC. We found that most of ferroptosis modulators displayed an association with each other. And the PPI network analysis showed that GLS2, SLC1A5, SLC7A11, GPX4, ALOX15, NFE2L2, CDKN1A, SAT1, ACSL4, and LPCAT3 had the potential to interplay with each other. These results indicated that these proteins potentially played their functions together and had similar functions in EC. Moreover, according to our analysis, we found that the expression levels of ATP5MC3, CDKN1A, SLC7A11, and SAT1 were related to the prognosis of EC. The higher expression level of CDKN1A, SLC7A11, and SAT1 resulted in longer DFS time. Nevertheless, highly expressed ATP5MC3 contributed to shorter DFS time in EC. Furthermore, our data suggested that high expression of SLC7A11, SAT1, and CDKN1A was linked to low the pTNM_stage, grade, and longer survival time. However, overexpression of TP53MC3 was linked to the advanced pTNM_stage, grade, and shorter survival time in EC. All the above-mentioned findings were in accordance with our previous analysis and indicated that SLC7A11, SAT1, and CDKN1A may serve as tumor suppressors and TP53MC3 may serve as an oncogene in EC.

The article "Identification of the Ferroptosis-Associated Gene Signature to Predict the Prognostic Status of Endometrial Carcinoma Patients" was published in 2021. Journal: Comput Math Methods Med.

These genes had been demonstrated as key regulators of ferroptosis and to function crucially in the development of carcinoma. SLC7A11 was firstly identified in 1980 by Bannai and Kitamura [43]. There has been a surge of reports demonstrating its pervasive expression in various cancers and multiple effects on cancer growth, invasion, metastasis, and unfavorable prognosis [43, 44]. For example, the progression of colorectal cancer stem cells could be specifically suppressed upon targeting SLC7A11, followed by inducing ferroptosis [45]. SLC7A11 was reported to confer resistance to ferroptosis in cancer cells and is adaptively expressed to reduce ferroptosis and buffer irradiation damages in lung cancer cells [46]. Overexpressing SLC7A11 promotes radioresistance in lung cancer cells through inhibiting irradiation-induced ferroptosis [47]. Suppressing the SLC7A11/glutathione axis resulted in synthetic lethality in lung adenocarcinoma with mutated KRAS [48]. The progression of non-small cell lung cancer was promoted by xCT- (SLC7A11-) mediated metabolic reprogramming. In this study, we found that SLC7A11, an attracting oncogene and an indication of an unsatisfactory prognostic status of liver cancer, was significantly downregulated in EC. Bioinformatics analysis showed that SLC7A11 was related to the regulation of multiple metabolism-related pathways and ERK activation. Overexpression of SAT1 brought about lipid peroxidation and ferroptosis under ROS stress [49]. SAT1 is a transcriptional target of p53 in human melanoma and lung carcinoma cell lines. Depleting SAT1 would hinder ferroptosis induced by p53 and p533KR. The polyamine catabolic enzyme SAT1 was responsible for the regulation of GBM tumorigenesis and the response to radiation [50]. Overexpressing SAT1 caused the apoptosis mediated by mitochondria in mammalian cells [51]. Here, our data suggested that EC highly expressed SAT1. Bioinformatics analysis showed that SLC7A11 was related to the regulation of multiple signaling, such as AKT phosphorylation of cytosolic targets, TP53 network, TAp63 pathway, hypoxia, and p53 in the cardiovascular system, cell cycle: G2/M checkpoint, and Notch signaling pathway, which demonstrated that this gene played a crucial role in EC progression.

The article "Identification of the Ferroptosis-Associated Gene Signature to Predict the Prognostic Status of Endometrial Carcinoma Patients" was published in 2021. Journal: Comput Math Methods Med.

Despite that immune checkpoint inhibitor (ICI) therapy has benefited some metastatic carcinoma patients, biomarkers needed for prediction are essential [52]. Some evidence from selected types of carcinomas suggested that TMB could be a predictor of clinical response to ICI [52]. Here, our study also aimed at evaluating the correlation between ferroptosis-related regulators and the TMB score in EC. The results depicted that ATP5MC3, CDKN1A, and SLC7A11 were significantly positively associated with the TMB score in EC. However, we did not observe a significant correlation between ferroptosis-related regulators and the TMB score in EC. These results implied that TP5MC3, CDKN1A, and SLC7A11 might serve as predictive markers of EC immunotherapy.

Also, we should point out several limitations of this study. First, most of the conclusions of this study were obtained using a single database, TCGA. Thus, more public datasets and clinical samples should be collected to further confirm our findings in this study. Second, the molecular functions of FRGs in EC remained to be further explored using gain or loss of function assay with siRNAs. Finally, only limited clinical information was available for us to perform bioinformatics analysis.

## 5. Conclusion

In brief, we identified that FRGs were significantly differently expressed in EC. Further analysis showed that SLC7A11, SAT1, CDKN1A, and TP5MC3 expression presented a negative relationship with the pTNM_stage, grade, and survival time. Bioinformatics analysis revealed that these genes participated in the regulation of cell cycle, citrate cycle (TCA cycle), metabolism-related pathways, ERK activation, p53 signaling pathway, cellular senescence, and Notch signaling pathway. It is worth noting that our data suggested that ATP5MC3, CDKN1A, and SLC7A11 were largely positively associated with the TMB score in EC. These findings for the first time showed that ferroptosis played a crucial role in EC.

## Figures and Tables

**Figure 1:** Gene expression of ferroptosis modulators in the development of EC. (a) The expression levels of HSPA, FANCD2, HSPB, CS, CARS, EMC2, TFRC, and SLC7A1 in grade 1, grade 2, and grade 3 EC and normal samples were shown. (b) The expression levels of NCOA4, GLS2, ACSL4, RPL8, GPX4, CDKN1A, LPCAT3, and NFE2L2 in grade 1, grade 2, and grade 3 EC and normal samples were shown. (c) The expression levels of DPP4, CISD1, SLC1A5, ALOX15, SAT1, FDFT1, and MT1G in grade 1, grade 2, and grade 3 EC and normal samples were shown. ^∗∗∗^*P* < 0.001 and ^∗∗^*P* < 0.01.

The article "Identification of the Ferroptosis-Associated Gene Signature to Predict the Prognostic Status of Endometrial Carcinoma Patients" was published in 2021. Journal: Comput Math Methods Med.

**Figure 2:** Identification of interaction among ferroptosis-related regulators in EC development. (a) The correlation among the expression levels of ferroptosis-related regulators in EC were analyzed using TCGA database. (b) The PPI network of ferroptosis modulators was constructed using the STRING database. ^∗∗∗^*P* < 0.001, ^∗∗^*P* < 0.01, and ^∗^*P* < 0.05.

**Figure 3:** Identification of DEFRGs associated with prognosis in EC development. (a–d) Higher expression levels of CDKN1A, SLC7A11, and SAT1 and lower expression of ATP5MC3 were related to longer DFS time. Nevertheless, highly expressed ATP5MC3 led to shorter DFS time in EC.

**Figure 4:** DEFRGs associated with DFS in EC development. (a–d) The median cutoff point of ATP5MC3, SAT1, SLC7A11, and CDKN1A, which was used to divide patients into the high-risk group and low-risk group. (e-h) The KM survival curves further showed the correlation between the expression levels of ATP5MC3, SAT1, SLC7A11, and CDKN1A and DFS time. (i–l) The area under the ROC curve (AUC) showed the predictive efficiency of CDKN1A, SLC7A11, SAT1, and ATP5MC3 in the 1-, 3-, and 5-year DFS.

**Figure 5:** DEFRGs associated with OS in EC development. (a–d) The median cutoff point of ATP5MC3, SAT1, SLC7A11, and CDKN1A, which was used to divide patients into the high-risk group and low-risk group. (e–h) The KM survival curves further showed the correlation between the expression levels of ATP5MC3, SAT1, SLC7A11, and CDKN1A and OS time. (i–l) The area under the ROC curve (AUC) showed the predictive efficiency of CDKN1A, SLC7A11, SAT1, and ATP5MC3 in the 1-, 3-, and 5-year OS.

**Figure 6:** The expression of ferroptosis-related regulators were related clinical characteristics in EC development. (a–d) SLC7A11, SAT1, CDKN1A, and TP53MC3 expression was differently expressed in EC compared to normal samples using GEPIA database. (a–d) We determined SLC7A11, SAT1, CDKN1A, and TP53MC3 expression and clinical characteristics in EC development, including the pTNM_stage, grade, and survival status.

**Figure 7:** The expression of ferroptosis-related regulators presented an association with TMB score in EC development. (a–d) The results showed the correlation between ATP5MC3, CDKN1A, SLC7A11, and SAT1 expression and TMB score in EC.

**Figure 8:** Bioinformatics analysis of ferroptosis-associated regulators in EC. (a–d) Bioinformatics analysis of ATP5MC3, SLC7A11, CDKN1A, and SAT1 in EC patients.

The article "Identification of the Ferroptosis-Associated Gene Signature to Predict the Prognostic Status of Endometrial Carcinoma Patients" was published in 2021. Journal: Comput Math Methods Med.

## Data Availability

All data generated or analyzed during this study are included in this published article.
